# Decision Tree Algorithm for Visual Art Design in a Psychotherapy System for College Students

**DOI:** 10.1155/2022/1255200

**Published:** 2022-07-14

**Authors:** Han Wang, Xiang Ji, Dandan Zhang

**Affiliations:** ^1^Academy of Fine Arts, Huaibei Normal University, Huaibei, Anhui 235000, China; ^2^College of Education, Huaibei Normal University, Huaibei, Anhui 235000, China; ^3^School of Computer Science and Technology, Huaibei Normal University, Huaibei, Anhui 235000, China

## Abstract

With the development of society, psychological health becomes a basic standard for a college student to grow into a qualified person. This study is aimed at using data mining principles and methods to excavate the factors that lead to psychological problems of college students, to purposefully carry out psychological interventions, use visual art design methods to promote college students' psychological health treatment, and build a perfect system of college students' psychological treatment. Based on the theories of data mining, we built a data analysis model, elaborated the data preprocessing method, and applied the Apriori algorithm to analyze the data of obsessive-compulsive symptoms and interpersonal sensitivity symptoms, and various psychological problem attributes extracted the strong association rules and analyzed the results. Take advantage of the corresponding unique school environment and educational advantages, to build a set of mental health education methods suitable for modern college students, and truly enable them to obtain satisfactory psychological interventions in a reasonable art design treatment phase. Based on the above association pattern mining results, a series of preprocessing operations were performed on the data, and then, the Apriori algorithm was applied to discover the potential association relationships among 9 psychological dimension factors of college students, and then, the ID3 decision tree algorithm was used to construct a decision tree and pruning process, from which the classification rules of students' psychological problems were analyzed and discovered. These studies provide some practical reference basis for school counseling work.

## 1. Introduction

The rapid development of the economy and the expansion of colleges and universities, as well as the consistent selection of talents by society, have made the competition between people more and more intense and consequently have led to a series of social problems. The psychological development of adolescents is not yet mature, and their ability to suffer setbacks and recover themselves is relatively weak. The formation of worldviews and values is not objective enough, and they are under the influence of various problems that can create great pressure and challenges, making adolescents a high-risk group prone to mental illness. With the growth of pressure in various aspects such as employment and examinations, students frequently commit suicide by jumping from buildings, which is heartbreaking and makes the whole society start to pay attention to the mental health of college students and start to think about how to make students have healthy psychology.

At present, all major universities have their psychological assessment systems, and they will generate and accumulate certain data after the psychological assessment work is finished every year, so the data accumulated year after year is increasing. After years of collection and convergence, the psychological assessment data become unique data resources; if not used for targeted analysis and utilization, it will only be dormant and worthless data and occupy hardware and software resources [1]. Therefore, it is necessary to obtain the important information hidden behind these data through certain technical means and to analyze and utilize these data at a higher level so that they can play their proper value. The existing psychological assessment systems generally have the functions of adding, deleting, modifying, counting, and querying data, but they cannot discover the valuable knowledge and laws hidden in the data, nor can they predict whether college students will have various serious psychological problems based on the existing data. The application of data mining technology can make up for this problem to a certain extent [2]. The decision tree algorithm has the features of high efficiency, easy to understand, small computation, good at handling discrete data, etc. Judging the goodness of a decision tree can be considered based on whether the decision tree is correct and whether it is more effective after passing the test of the sample data set and its complexity, indirection, and scale. After years of use, the college counseling system has accumulated a large amount of students' psychological assessment data, and if the relevant technology and algorithm of data mining can be used for mining, it is very likely to understand the causes of students' problems at a deep level. For this purpose, it is necessary to discover the existing accumulated large amount of student psychological assessment data [3].

This paper takes the psychological assessment data of college students as the data mining object and then applies the association rule algorithm and decision tree algorithm to the research object, in turn, to construct the corresponding mining model and decision tree, and then analyze the key factors leading to the psychological problems of college students. The mining results of the two algorithms were combined and fed back to the counselors for better psychological intervention and guidance.

A decision tree is a tree structure that includes three parts: root node, branches, and leaves. The root node represents an attribute of the tree, the leaves represent the tokens of the classification, and the branches represent the output results [4]. The method iterates iteratively from the root node and assigns instances to its children based on the results obtained from the test; each child node corresponds to a value taken for that feature and continues to test and assign instances through a recursive method until it reaches the leaf node and finally assigns instances to the class of the leaf node. In the decision tree, there are two kinds of data sets: sample data set and test data set. The sample data set is a collection of data in which the attributes and classifications are known, and the algorithm is used to train the sample data set and finally produce the corresponding decision tree. The test dataset is used to test the generated decision tree, bring the data into the decision tree, derive the final categories, compare it with the actual types, and measure the accuracy of the decision tree [5]. The decision tree algorithm has the features of high efficiency, easy to understand, small computation, good at handling discrete data, etc. To improve the accuracy and efficiency of subsequent mining, data preprocessing is required beforehand. Data preprocessing is a key aspect and important step in data mining. Transforming data, summarizing and reducing data, cleaning data, and integrating data are several methods commonly used for data preprocessing. A decision tree can be judged based on whether it is correct and whether it is more effective after passing the test on the sample dataset and its complexity, indirection, and scale.

Mental health education is also a process of gradual establishment and expansion, from the beginning of courses and educational lectures on psychology and mental health, holding mental health competitions, carrying out some scientific work on mental health knowledge, to the establishment of full-time counseling rooms in schools. In recent years, with the development of science and technology, especially the development of computer science and technology, there are various assessment websites on the Internet [6]. Schools have also started to develop assessment websites where students can take assessments online and the websites will analyze individual and group behavioral characteristics to give appropriate results and suggestions based on the results of the assessments.

Art therapy, also known as art psychotherapy, is one of the psychotherapies. The synthesis of psychodiagnostic and artistic disciplines is accomplished through the media of art design, dance, drama, poetry, and visual arts. The patient's artistic creation is not only a way of self-expression but the finished product is considered one of the important diagnostic tools, based on psychotherapeutic theories and methods, which help to alleviate psychological problems and promote psychological well-being, based on the physiological and psychological effects of the visitor's activity in the arts. The visual effect depends on the interaction between the two sets of correspondences: the visual subject and the visual object, and the visual perception arises from the interaction of these two sets of relations. This way of thinking is determined by the patient's physiological characteristics, and once this process of action forms a thinking orientation, it will play a role in the mental adjustment of the perceptual process of visual perception [7]. When visual perception and thinking judgments are in agreement, a sense of empathy and pleasure is generated. Similarly, if the visual perception and the thinking judgment feel different, the visual perception will produce a sense of resistance and discomfort to the logo design, which is the dynamic nature of visual perception. Therefore, when designers design the logo design, they should take into account the patient's visual perceptual feelings and have a full understanding of the process of mutual verification and visual integration between the patient's feelings and objective forms to make the logo design truly “vision-based.”

Physical needs are the most primitive and basic needs of patients; they have the significance of maintaining personal survival and racial protection, and it is the basis for generating other needs. The need for safety refers to the need for people to remain stable, acceptable, and free from threats in their lives. Social needs refer to the needs of friends and family and the need for acceptance and recognition by surrounding groups and organizations [8]. The need for respect refers to the patient's quest for respect and worth, including self-esteem and respect. The need for self-fulfillment refers to the desire to accomplish things that are commensurate with one's abilities. The need for self-fulfillment begins with a layer-by-layer satisfaction of the patient's needs. The intensity of the various needs will vary in different environments and at different times, and there is always one in the dominant position. Similarly, in the process of logo design, attention should be paid to the needs of patients at different levels, taking into account the physiological characteristics and psychological needs of patients, to make a reasonable expression of the design form with a target, from the starting point of satisfying the needs of patients, so that patients and logo design form a good interactive relationship, which is conducive to the recovery of their diseases.

## 2. Method

### 2.1. Design

At present, most of the psychological assessment systems do not have a data mining module, and the role of the system is limited to data collection and simple statistical analysis, without the function of analyzing the potential relationship between each attribute of student information and various psychological symptoms, and there is no reliable basis for college counselors or psychological counselors to carry out preventive interventions; therefore, this makes the application of data mining techniques to college psychological assessment data is called the need and necessity [9]. In this chapter, the association rule mining algorithm is applied to the psychological assessment data of college students for research.

The process of data mining is different in different areas of expertise. Each data mining technique has its different characteristics and implementation steps. Therefore, the data mining process also varies for different needs, such as data integrity and professional support, which can have an impact on the mining process, and this leads to differences in data mining and the overall planning process in different regions. Even within the same industry, there are significant differences due to different analytical techniques combining different levels of expertise. Before data mining can be implemented, it is important to determine the steps to be used, what is to be done at each step and what is to be achieved. There must be a well-thought-out plan for data mining to be implemented in an orderly manner and be successful. Many software vendors and data mining companies provide users with several data mining process models to guide these users step-by-step through data mining [10]. The data mining process based on the decision tree algorithm in this paper mainly includes several stages as shown in Figure 1.

The normalized Gini coefficient is the product of the Gini coefficient of a child node and the ratio of that node to its parent node, so the larger the Gini coefficient, the greater the uncertainty, i.e., the greater the impurity, when *D* is divided by *A*. CART can produce both discrete results, which are discrete results, and continuous results, which are regression results. The created tree is also called a regression tree. To obtain regression results, it is useful to use the numerical analysis methods of LSD and LAD to process the data samples, which are useful in regression trees.

### 2.2. Dataset

The whole process starts with the acquisition of the data source, which is the data preparation work. The raw data is extracted from the psychometric system, and the raw data is generated by logging in to the system by the administrator and logging in to the system by the students. First, the administrator logs into the psychological assessment system to import various assessment questionnaires, including the SCL-90, which can be added, deleted, and modified by the administrator, and then, the counseling center administrator organizes students to fill out the SCL-90 form on the computer room and improve their personal information so that the information is stored in the database of the psychological assessment system [11].

The present study used the data of the results of the SCL-90 symptom self-assessment scale of the current cohort of students as the research object, used the association Apriori algorithm to mine the association rules for each psychological factor, and used the decision tree algorithm in the classification to mine the implied relationship between each attribute in the basic information of the students and the psychological symptoms with a high probability of occurrence, and then analyzed the obtained rules.

### 2.3. Data Preprocessing

High-quality data mining results come from high-quality data. The three elements of data quality are accuracy, completeness, and consistency. The raw data we obtain in reality usually have problems such as inconsistency, duplication, containing noise, and high dimensionality. To solve these problems and improve the accuracy and efficiency of subsequent mining, data preprocessing is needed beforehand. Data preprocessing is the key link and important step in data mining; transforming data, summarizing and reducing data, cleaning data, and integrating data are several common methods of data preprocessing. When conducting the design of signage design in art therapy centers, it is important to consider the laws of perception of images and the preferences and laws of different colors of patients with psychological disorders. Therefore, it is not wrong to pay attention to the needs of patients and design from their point of view in the logo design of art therapy centers. Among them, data cleaning can be used to remove the noise present in the data and correct the inconsistency problem; data set can merge data from multiple data sources into a complete and consistent data store; data transformation can compress the data to a smaller interval, thus contributing to the efficiency of mining algorithms using distance metrics and the accuracy of the executed results; remove redundant data by clustering and reduce data size by clustering [12]. The various data preprocessing methods described earlier can be used simultaneously or selectively, to obtain high-quality data after professional and scientific processing, thus preparing for high-quality mining results and thus producing good decisions.

### 2.4. Data Normalization Process

The SCL-90 scale corresponds to three levels of symptoms: mild, moderate, and severe. Symptoms with a score of not less than 4 are considered severe, those with a score greater than or equal to 3 and less than 4 are considered moderate, and those with a score less than 3 are considered mild. According to the statistics, the proportion of students with severe symptoms in each dimension is generally less than 0.1%. If a high threshold of minimum support is set, frequent items are often filtered out in the process of mining the frequent itemset because the support of the lower frequency items is less than the minimum support threshold. Therefore, in this paper, we use “yes” and “no” to distinguish the symptoms of each dimension and binarize “yes” with 1 (score ≥ 2) and “no” with 0 (score < 2), since we use 3000 yuan as the cut-off point to get the number of people in the two intervals. Since the difference between the number of people in the two intervals is not large, the continuous data “monthly household income” is discretized into two intervals, high and low, by using 3000 yuan as the cut-off point. The high interval corresponds to ≥3000 yuan and is represented by the number SR1 [13]. The low interval corresponds to ≤3000 yuan and is represented by the number SR0; “where did you live since childhood” is also discrete data, in which rural and small towns are generalized to rural areas and large cities and foreign countries are generalized to cities so that only rural and urban areas remain after generalization, and the corresponding numbers are SZD0 and SZD1. For the attribute of whether or not they grew up with their parents, option A is set to yes, while the other options of growing up with friends and relatives, grandparents, and others are set to no, corresponding to the numbers GW1 and GW0, respectively. For the attribute of whether both parents are alive or not, option A is set to yes, and the corresponding number is SQ1; other options such as divorced and remarried, both parents are dead and divorced and single are all types of missing parents, so they are set to no, and the corresponding number is SQ0, as shown in Table 1.

Each transaction in the above dataset contains 6 basic student information attributes and 9 psychological dimension factors, i.e., corresponding to the psychometric symptom data of a tested student and the student's attributes. Each subset contains 6 attributes and one type of psychological dimension factor. The decision tree is a top-down recursive division, which uses a top-down, divide and conquer approach, and its basic algorithm is essentially greedy [14]. Starting from the root node, each non-“leaf node” is found to have an attribute in its corresponding sample set to test the sample set, and the training sample set is divided into several subsample sets according to the different results of the test. Each subsample set constitutes a new “leaf node,” and the above process is repeated for the new “leaf node” so that the cycle continues to a specific termination condition. The key aspects of building a decision tree are how to divide the sample set and the selection of test attributes. Different techniques are used in different decision tree algorithms. The decision tree uses a top-down recursive approach to compare and evaluate the attribute values of the nodes inside the decision tree and to determine the branching from the node down according to the different attribute values.

### 2.5. Results

The attributes in the dataset selected for this paper all have only two attribute values, so the disadvantage of the ID3 algorithm which tends to select multiattribute value attributes is circumvented. ID3 algorithm is a traditional decision tree construction algorithm that selects the optimal split node by calculating the information gain of each attribute and then comparing the size. Therefore, it was decided to use the ID3 algorithm for the classification mining of student psychological problem data.

In this paper, we first preprocess the original data set; then randomly select two-thirds of the preprocessed data set, about 5384 records, as the training sample set; construct a decision tree based on the ID3 algorithm; and use the remaining 2691 records as the test sample set to test the decision tree constructed using the training set. Facing the scenario of high-dimensional data, the Diff-PCCDT algorithm proposed in this paper and its parallel implementation of DiffMR-PCCDT may be powerless. Therefore, in future work, we can consider adding corresponding modules to this algorithm to handle high-dimensional data to further improve the efficiency and usability of the algorithm. The detailed steps for constructing a decision tree model for students with or without obsessive-compulsive symptoms using the ID3 algorithm are as follows: first, the information gain of each splitting attribute in the training sample set is calculated using equations (4.1), (4.2), and (4.3). Then, the information gains generated according to different split attributes are compared, and the attribute with the highest information gain is set as the root node of the decision tree, and then, the number of branches generated downward according to the number of values of this attribute at this root node is determined, and also, the total training sample is divided into several subdatasets [15]. Finally, the first two steps are performed recursively on each split subdataset until the leaf node of the spanning tree or no attribute is available for further splitting; then, it ends. The training sample set *D* is randomly selected, according to which we can learn that the attribute QP (obsessive-compulsive symptom) has two different values: 0 (no symptom) and 1 (symptomatic) [16]. Therefore, the training sample set can be divided into two categories, which there are 1162 samples with the value of “1” and 4222 samples with the value of “0.”

According to the formula *K*_*ρ*_(*x*, *y*) = *φ*∑_*y*∈*γ*_∑_*x*∈*χ*_[*p*(*x*, *y*) · ln*p*(*x*, *y*) + *Ax* + *Cy*] + *λ*, the expected information of the training sample *D* classification, i.e., the entropy, is calculated as *K*_*ρ*_ = 0.7839. Next, the entropy of each split attribute needs to be calculated. Taking the gender attribute as an example, there are 2170 items with gender as male (XB1), among which 450 are symptomatic and 1720 are asymptomatic; there are 3214 items with gender as female (XB0), among which 712 are symptomatic and 2502 are asymptomatic.

### 2.6. Analysis

For discontinuous data, generalization techniques are usually applied to process them, while continuous data are processed by discrete processing in this paper. That is, continuous data is artificially divided into several reasonable intervals, set an interval line to represent the individual data summary values, and calculate a specific discrete symbol expressed in this interval range, usually with two steps: determine the segmentation of discrete points and statistical or description of the segmentation interval [17]. After years of collecting and aggregating psychometric data, it becomes a unique data resource, and if it is not used for targeted analysis and utilization, it will only be dormant and worthless data and occupy software and hardware resources. It is well known that patients undergoing art therapy are part of a special group that differs from ordinary patients with diseases in terms of psychological and physiological aspects as well as in their response to external stimuli. Therefore, when carrying out the design of signage design in art therapy centers, it is necessary to consider the rules of perception of images and the preferences and rules of different colors of patients with psychological disorders. Therefore, it is not wrong to pay attention to the needs of patients and design from their point of view in the logo design of art therapy centers.

Based on the visual perceptual characteristics and safety needs of patients with psychological disorders, patients with psychological disorders need designs that bring a relaxing psychological effect. When patients with psychological disorders are perceiving the objective world, the simplified transmission of forms will make it easier for patients in a period of unstable thinking and logic to understand and recall more easily, and it is a good visual effect to feel the inner sense of relaxation from the appearance of form expression. At the same time, it also makes patients relax their vigilance, so in the logo design, the first thing is to give patients a simplified feeling visually and arrange all the elements appearing in the picture based on this principle. The simplification of logo design is to incorporate color graphics in the appropriate form to communicate the design, which is also pleasing visual imagery [18]. The transmission of such a feeling is stimulated by the visual form, prompting the psychological and thinking active process, a collection of various forms of simplification of expression and the visual effect.

## 3. Results

### 3.1. Sample Selection

This experiment adopts its own controlled experimental scheme to systematically design and establish a psychological prevention and intervention program suitable for mental health education research in colleges and universities, as well as to establish the necessary operational mechanism and evaluation system in participatory intervention activities. At the same time, while serving college students, this project explores an effective localized resource integration and utilization mechanism to transform the research results into a suitable mental health service model; in the process of establishing, implementing, maintaining, and updating the model, it can promote the professional quality and cultivation of the participants, which is both the purpose of the study and the advancedness of the method; it is both a survey study and a prospective study and a pioneering work. All were subjected to a preintervention assessment questionnaire for the target population before enrollment, and several counselors were treated with a case-based intervention. As shown in Table 2, all the data before and after treatment were significantly lower than the scores before treatment, including depression from 1.71 to 1.63 and paranoia from 1.68 to 1.59.

The MR-PCCDT algorithm is mainly based on the nonparallel algorithm PCCDT, which employs the MapReduce parallel framework in its split phase to enable it to efficiently process large data sets and therefore also has the described privacy issues. Now assume that the MR-PCCDT algorithm is running in a cloud computing scenario. This scenario consists of three main entities: (1) the data owner, which owns a large dataset and allows organizations or individuals to run the MR-PCCDT algorithm on the dataset to query it to obtain useful results; (2) a service provider, which provides the entire computing environment and allows the data owner to share and upload data while allowing institutions or individuals to run MR-PCCDT algorithms on this data to query it; and (3) organizations or individuals who want to run MR-PCCDT algorithms on the shared and uploaded data to achieve their goals and who may maliciously infer data to find some private information they want to know [19].

### 3.2. Experimental Results and Analysis

By comparing the results produced on the datasets Adult and Mushroom, we can see that the algorithm DiffMR-PCCDT is not more accurate than the algorithm Diff-PCCDT when tested on clusters with different numbers of nodes, although the difference between the two algorithms is small [20–22]. This is because the algorithm DiffMR-PCCDT is not the same as Diff-PCCDT, so there is a slight difference in performance. However, this paper can also roughly conclude that the performance of the two algorithms is similar in terms of tested accuracy on the classification problem. In addition, some comparisons are made on larger datasets (e.g., Skin, Cover type, and KDD Cup) with sample sizes of 245,057, 581,012, and 494,021, respectively, on which the nonparallel algorithm Diff-PCCDT is attempted. Unfortunately, the experiment was terminated because the run time for the dataset Skin exceeded 48 hours and memory warnings occurred on the other two datasets. Data cleaning can be used to remove noise from data and correct inconsistency problems; datasets can combine data from multiple data sources into a complete and consistent data store; data transformation can compress data into smaller intervals, thus facilitating the efficiency of mining algorithms using distance metrics and the accuracy of the execution results; removing redundant attributes by aggregation and reducing the size of data by clustering are both methods used for data imputation. The results from the comparison of these three large datasets show that the parallel algorithm DiffMR-PCCDT can effectively solve the time complexity and memory limitation problems, which often occur in traditional nonparallel differential privacy decision tree algorithms for big data classification problems, as shown in Table 3.

The paper then tests the runtime differences between the algorithms DiffMR-PCCDT and Diff-PCCDT on the Adult, Mushroom, EEG eye, Electricity, Magic, and Nursery datasets. The comparison results are shown in Figure 2, from which we can draw two conclusions [23]. One is that the parallel algorithm DiffMR-PCCDT can significantly reduce the runtime compared to the nonparallel algorithm Diff-PCCDT. The other is that as the number of nodes in the cluster increases slightly, the runtime of the parallel algorithm DiffMR-PCCDT tends to decrease.

The proposed parallel algorithm DiffMR-PCCDT is validated in terms of test accuracy and runtime on nine medium-large datasets with a different number of nodes [24]. By comparing with the nonparallel algorithm Diff-PCCDT, this chapter concludes that DiffMR-PCCDT is comparable to Diff-PCCDT in terms of test accuracy, but the former is significantly better than the latter in terms of runtime. The experimental results demonstrate the feasibility of the DiffMR-PCCDT algorithm, which can ensure the testing accuracy and running efficiency of the algorithm while satisfying differential privacy protection and is suitable for practical application scenarios.

Some companies or individuals can find a lot of valuable information by analyzing and mining the collected personal data. Pearson correlation coefficient-based decision tree (PCCDT) as a new type of decision tree algorithm has been widely used in many fields, such as pattern recognition, machine learning, and information retrieval [25]. However, when the dataset contains sensitive personal information (e.g., patient's diagnosis information and customer's shopping information), mining and analyzing the dataset using Pearson correlation coefficient-based decision trees may create privacy leakage problems, which may threaten the privacy security of users. Based on the Pearson correlation coefficient-based decision tree algorithm, we propose a Pearson correlation coefficient-based differential privacy decision tree algorithm to ensure the effectiveness and usability of the algorithm while satisfying the differential privacy [26].

### 3.3. Calculate Information Gain

The information gain is the category information entropy of the dataset—the conditional entropy of each classification. The higher value of information gain is calculated; it means that the samples classified according to this attribute can reduce the uncertainty of the classified samples, so the selection of this attribute as the classification attribute of the node can be associated with the better accomplishment of the classification goal. In the ID3 algorithm, information gain is the indicator of feature selection [27]. The intuitive meaning of information gain is the reduction of uncertainty after the label is divided by the attribute. If we simply use information gain as the judgment criterion, we can imagine that when a certain attribute has many values, the label will be divided into many copies, so its uncertainty will naturally be reduced a lot, and then, the ID3 algorithm will prefer to choose this attribute as the basis for classification, which is not what we want. Therefore, C4.5 chooses to improve ID3 by using the information gain rate [28–30]. The intrinsic information of an attribute refers to the information about the number and size of branches when a certain attribute is divided using the division information metric to be considered. According to the information gain/intrinsic information of an attribute, it is possible to make the importance of an attribute decrease as the intrinsic information increases, which means that if the uncertainty of an attribute is greater, the less inclined it is to be selected. It compensates for the pure selection of information gained as a feature selection index [31].

## 4. Discussion

In this study, the accuracy of the remaining one-third of the data was validated by applying it to the generated decision tree classification model, where the status of the remaining data in terms of obsessive-compulsive symptoms was already known, and using the initially generated decision tree to predict the classification of the test set, the already existing categories were compared to the predicted classification results with an accuracy of 73%; the predicted classification results of the test data set using the pruned decision tree were compared. The accuracy was 79.6% when comparing the predicted classification results of the test data set with the known categories [32–34]. For discontinuous data, we usually apply generalization techniques to process them, while continuous data are processed by discrete processing in this paper. That is, continuous data is artificially divided into several reasonable intervals; an interval line is set to represent each data summary value, and a specific discrete symbol is calculated to express this interval range. Therefore, it is evident that the results of classification mining of psychometric data by using the ID3 decision tree algorithm to construct decision trees and pruning based on the PEP algorithm can be useful for psychological prevention and intervention. Based on the introduction of the splitting rules for constructing decision trees, the process of constructing decision trees based on the ID3 algorithm is described in detail, followed by the postpruning process of the decision trees using the PEP pruning leaf algorithm, and finally the analysis of the resulting classification rules.

## 5. Advantages and Limitations

Apriori algorithm and decision tree ID3 algorithm are used in this study, and the research method of applying the two algorithms to predict the psychological problems of college students is described. However, due to the limitation of time and own level, there are some shortcomings and deficiencies in the research of data mining in mental health management system in this paper, and many of the research ideas are not all completed in the paper, and we hope that some of the remaining problems can be further studied in the future when the conditions allow [35]. It is possible to study the integrated development of functional modules for data mining so that the psychological assessment system not only has information collection and general statistical functions but also can have functions such as correlation prediction processing using data mining core algorithms, expanding the functional means of psychological problem analysis. The method used for data preprocessing is slightly simple, and the constant substitution method is used for some small amount of null values in the data source; i.e., the missing values and more diversified data cleaning strategies can be tried in practical applications.

The signs of art therapy center serve actors in design form. When expressing the visual effect, the process of constructing the signage design in art therapy centers should take into full consideration [36]. The visual effect should be taken into account the psychological and physiological characteristics of the audience, and create psychological harmony for patients as much as possible, so as to surpass physical harmony. When all these design forms are satisfied, patients with psychological disorders will be able to feel better in the environment [37]. When these design forms are satisfied, patients with mental disorders will have a better feeling in the environment for treatment, which is conducive to the recovery of their illness.

## 6. Future Research Directions

This paper focuses on the privacy problem of the Pearson correlation coefficient-based decision tree algorithm, proposes a Pearson correlation coefficient-based differential privacy decision tree algorithm Diff-PCCDT and its parallel implementation DiffMR-PCCDT in the MapReduce framework, and builds a college student heart health treatment system by combining the artistic design approach [38]. Theoretical analysis proves that both the proposed Diff-PCCDT algorithm and DiffMR-PCCDT algorithm satisfy the differential privacy requirement. By comparing with the classical differential privacy decision tree algorithm DiffP-ID3 on several small- and medium-sized datasets, the experimental results show that Diff-PCCDT outperforms the DiffP-ID3 algorithm in terms of overall testing accuracy [39]. In addition, a comparison of the parallel algorithm DiffMR-PCCDT with the Diff-PCCDT algorithm on several media to large datasets verifies its effectiveness and good operational efficiency. (1) The proposed Diff-PCCDT algorithm and its parallel implementation DiffMR-PCCDT may not be able to cope with the scenario of high-dimensional data. Therefore, in future work, we can consider adding corresponding modules to the algorithm to deal with high-dimensional data to further improve the efficiency and usability of the algorithm. (2) For the parallel algorithm DiffMR-PCCDT that processes large data, the privacy budget may be tight in the case of satisfying differential privacy, because the larger the dataset may lead to consuming more privacy budget. How to design a better privacy budget allocation scheme to reduce the consumption of privacy budget can be a future research direction.

## 7. Conclusion

This paper takes the psychological assessment data of a university as the data mining object and then applies the association rule algorithm and decision tree algorithm to the research object, in turn, to construct the corresponding mining model and decision tree, and then analyze the key factors leading to the psychological problems of college students. By taking students' social anxiety and depression as the entry point and designing the treatment with the help of art, we can reasonably improve and enhance the mental health of college students and synthesize the results of the two algorithms to feedback to the counselors for better psychological intervention and guidance effectiveness. The results of the two algorithms are combined and fed back to the counselors for better psychological intervention and guidance. From the perspective of college students' mental health education, this paper comprehensively explains the importance of art and design therapy for adjusting students' bad emotions, fully utilizing the modern art and design therapy, based on the principles and mechanisms of art and design therapy, and under the premise of analyzing the psychological conditions of modern college students, using the corresponding unique advantages of the school environment and education, to build a set of mental health education suitable for modern college students. In addition, through our own practical experience and active exploration and exploration, we can build a reasonable and perfect art design therapy system.

## Figures and Tables

**Figure 1:** Number mining process based on decision tree algorithm.

**Figure 2:** Running times of the algorithms DiffMR-PCCDT and Diff-PCCDT on several datasets.

**Table 1:** Table contents after conversion.

XB	GK	SR	SPL	SL	QUH	CP	LKMO	PCE	LM
XB0	GK0	SR1	SPL2	SL0	0	1	0	1	2
XB1	GK1	SR0	SPL1	SL2	1	0	1	0	0
XB2	GK2	SR2	SPL0	SL1	0	2	1	1	1
XB3	GK4	SR5	SPL3	SL6	1	0	1	0	0
XB4	GK7	SR3	SPL6	SL4	2	1	2	2	2
XB5	GK3	SR7	SPL7	SL7	0	0	2	1	0
XB6	GK6	SR4	SPL5	SL5	1	2	1	0	1
XB7	GK5	SR3	SPL4	SL3	1	1	0	2	1

**Table 2:** Pre- and posttreatment comparison of depression.

Evaluation factors	Before	After	*t*
Depression	1.71	1.63	2.492
Paranoia	1.68	1.59	3.423
Fear	1.93	1.86	3.245
Anxiety	1.68	1.52	2.543
Aggressiveness	1.83	1.75	3.124
Sensitive	1.47	1.42	2.353

**Table 3:** Test accuracy of the algorithms DiffMR-PCCDT and Diff-PCCDT on medium and large datasets.

Dataset	DiffMR-PCCDT	Diff-PCCDT
Adult	1.9302	1.8904
Mushroom	0.9334	1.3492
EEG eye	0.8941	1.2091
Electricity	1.2803	1.3942
Magic	1.3094	1.5321
Nursery	0.9482	0.9723

## Data Availability

The data used to support the findings of this study are available from the corresponding author upon request.
